# Recognition and Optimization Analysis of Urban Public Sports Facilities Based on Intelligent Image Processing

**DOI:** 10.1155/2021/8948248

**Published:** 2021-12-02

**Authors:** Hao Li, Dujuan Li

**Affiliations:** Department of Physical Education, North Sichuan Medical College, Nanchong, Sichuan 637000, China

## Abstract

In the utilization of urban public facilities, it is found that the number of people under 18 years who exercise accounts for 29.5% of the total number of people surveyed, 32.8% between 18 and 65 years, and 37.7% over 65 years. The elderly have become the main population of public facilities, and the aging of cities is becoming more and more obvious. Strengthening the construction and development of urban public facilities has become the main work of current urban construction, and planning public facilities can effectively alleviate the pressure of urban public facilities. Through image recognition to promote urban sports public service, we improve the management efficiency of urban sports public service, facilitate residents' sports, and improve residents' satisfaction and happiness index. Through image recognition to manage portraits and objects, the safety of residents' sports and sports facilities is guaranteed, and the management efficiency is improved. The experimental results show that R-CNN, FAST R-CNN, and Faster R-CNN in urban public facilities can be intelligently recognized by image recognition technology for comparison. Faster R-CNN has good accuracy and low average time. Finally, the study analyzes the service cost of public facilities, compared with traditional public services, with the application of public services under image recognition, so as to guide different groups of people to make full use of public service facilities to improve their quality of life and realize the good behavior of the national movement.

## 1. Introduction

With the development of the times, in order to improve people's sports satisfaction index, sports facilities can be managed through urban sports public services under image recognition. Using image recognition and DEA model and SE-DEA model for public service efficiency management to improve management efficiency, we create a safer and more comfortable sports experience, meet the needs of residents for physical exercise, improve the safety and comfort of sports facilities, carry out sports activities in schools, enterprises, and communities, improve public sports awareness, and better develop urban public services through image recognition.

In [1], photos of viewers in activities are extracted for information identification and output through a systematic method of photographic equipment and multiple viewers were associated with individuals. Shih et al. [2] identify adult images by image retrieval technology and retrieve 100 images from adult and nonadult galleries based on feature tests such as pigment. If the retrieved images contain multiple adult images, they are regarded as adult images. Through this method, children are prevented from contacting pornographic content through browsers in the era of developed Internet. Takeda et al. [3] verify identity in less than 0.1 seconds by finger image recognition. This method is based on the whole finger image and finger joint line pattern. This method is not disturbed by external factors, low cost, and simple algorithm; through experiments, the experimental error rate is low. Kousha et al. [4] discuss whether a large number of digital pictures in the network are copied or reused on the Internet of Things to evaluate the influence of science or art. Although it is reasonable to judge the value of image reuse from TinEye's data, the scope of reference is unclear. Ruiz-Llata et al. [5] show that the vision system is realized by neural network processor prototype of discrete optical and photoelectric devices through experiments and describe the realization of neural network processor prototype system. In [6], through the analysis of the development of urban sports public services in China, we know that there are drawbacks in the supply of urban sports public services in China. No corresponding complete system of urban sports public service has been formed. The reason lies in the coordination between the government and the market. The main factors include insufficient resources and sites, low utilization rate, and inadequate supervision of facilities management. The coordination between government and market is strengthened. In [7], by establishing urban and rural sports public service management system, improving the coverage rate of sports public service in cities and villages, expanding the coverage area of venues, rationally planning sports public service, and training professional teams, the coverage rate and policies of sports public service in six cities of Jiangsu Province can be improved. The management system of sports public service is promoted in six cities of Jiangsu Province. Lu et al. [8] strengthen the formulation of the integration of urban and rural sports public services and the training of relevant professionals, supervise and manage urban and rural sports public services, and strive to develop the integration of urban and rural sports public services. In [9], through research, we know that there are some defects in the current sports public service, flaws in the mechanism management, and people's weak awareness of physical exercise. In order to create better urban sports public service facilities, with the development of the times [10], people have higher requirements for sports public service facilities. In order to meet the relevant requirements, the quality and management level of urban sports public services should be improved. Zhang [11] puts forward the combination of field programmable gate array (FPGA) and convolution neural network (CNN) and obtains a new concept of sports, which made urban and rural sports public services develop together and improve satisfaction. In [12], the development of social economy is closely related to urban community public services. The development of urban sports public services should adhere to the principle of equality, and the sports services of villages and towns and cities should be developed in a unified way. In [13], during the social transformation, the development of urban sports public services in China is uneven with that of country and town sports public services. It is necessary to fundamentally improve this flaw. Liang [14] compares the differences of sports public services between urban and rural areas in Beijing by various methods, as well as the investment and development of public facilities and the participation of residents in physical fitness. In [8], the integration of urban and rural sports public services includes the formulation and application of policies, among which the integration of the policy system is the most important component and the management policy of public services is strengthened. In the above research, the existing policy problems or the low accuracy of the analysis algorithm are analyzed from the perspective of urban public facilities. However, as the influence of population, gender, age, educational level, and other factors has an impact on the current situation of urban sports, using image recognition technology can improve the utilization rate of the corresponding public facilities and can analyze the planning and effective utilization of public facilities.

## 2. Understanding of Urban Sports Public Service under Image Recognition

### 2.1. Understanding of Image Recognition

The image recognition [15–17] flowchart is shown in Figure 1. Its advantages are as follows. Noncontact: users do not directly contact the equipment. Optional: face recognition [18] can be used to obtain information in advance. Parallelism: multiface contrast and shooting can be carried out at the same time. Item ID can be used for self-service, photo purchase, and identification of the same item in Figure 1.

The specific process of face recognition is shown in Figure 2.

The detailed process of fingerprint identification is shown in Figure 3.

Fingerprint identification process is divided into two secondary processes, which are divided into four parts. Two secondary processes are fingerprint recording and cross checking.

Fingerprint recording process consists of four parts: fingerprint collection, fingerprint preprocessing, fingerprint inspection, and fingerprint template collection.

Fingerprint comparison process also includes four parts: fingerprint collection, fingerprint preprocessing, fingerprint feature comparison, and matching.

In these two processes, the preprocessing of fingerprint image exists, but the value of the fingerprint image and the value of fingerprint feature seem to have the same name, but their inherent algorithms and properties are completely different.

In the process of introducing fingerprints, fingerprint images are obtained more frequently, while the single-value extraction algorithm pays more attention to the discrimination and acquisition of some eigenvalues.

### 2.2. Urban Sports Public Service Planning

In order to promote urban residents' sports and physical exercise, improvements should be made from the following aspects:

1. Strengthen the construction of sports public facilities in poverty-stricken and border areas, enhance the concept of urban sports public services, and make the elderly and young people in remote and poverty-stricken areas understand the necessity and importance of sports. Realize the popularization and all-round development of sports public services.
2. Strengthen the management of urban sports public services. Formulate strict management regulations, train professional management talents, popularize relevant sports methods, and reduce sports injuries. Repair sports venues and facilities, and open them to the outside world. Make everyone have sports rights and sports venues. Manage the safety of facilities and sites through security personnel.
3. Accelerate the popularization of sports, and make urban residents participate in sports and experience the fun of exercise through community, enterprise, and school sports meetings, so as to improve their interest in sports and their satisfaction with sports public services.
4. Actively promote sports, actively publicize the benefits of sports through performances and dissemination of sports knowledge, and ensure residents' sports and participation.

Divide sports facilities into public and private ones. Its structure is as shown in Figures 4 and 5.

The specific planning of urban sports public facilities is shown in Figures 6 and 7.

The quality of sports public service is affected by many factors. In order to bring better experience of urban sports public service to residents, we should conduct in-depth exploration and management according to many factors, improve the management quality of urban experience public service, bring better experience of sports to residents, and create the wind direction of national fitness.

### 2.3. Utilization of Urban Sports Public Service

#### 2.3.1. Necessity of Urban Sports Public Service Construction

1. Cultivate competitiveness through competitive sports. Through competitive training, people are more motivated.
2. Train athletes through physical education. The strength of athletes shows the physical health of people in a country. Only when people's physical fitness is enhanced can they work and go to school better.
3. Ensure the normal use of sports management. Evacuation passages are posted in the gymnasium to prevent accidents and emergencies, and safety evacuation drills are conducted regularly in the gymnasium to prevent travel accidents when accidents occur.

#### 2.3.2. Utilization of Social Resources by Urban Sports Public Service

1. Vigorously develop the construction of local sports venues and facilities such as schools, communities, and companies through the government, enterprises, and schools. Relieve the financial pressure through government investment.
2. Introduce market-oriented management and marketing. The gymnasium is built in the city center, which is convenient for residents to use.
3. Ensure the safety and usability of the gymnasium. Evacuation passages are posted in the gymnasium to prevent accidents and emergencies, and safety evacuation drills are conducted regularly in the gymnasium to prevent travel accidents when accidents occur in Figure 8.

## 3. Analysis on the Present Situation of Urban Sports Public Service

### 3.1. Mediation Effect and Chain Mediation Effect Model

Improve the efficiency of public service [19] through this algorithm in Figure 9.where ABC is the regression coefficient.

(1) $$\begin{array}{c} Y=cX+\varepsilon_{1},\\ M=aX+\varepsilon_{2},\\ Y=c^{\prime }X+bM+\varepsilon_{3}, \end{array}$$

### 3.2. Improve the Effectiveness through DEA Algorithm

#### 3.2.1. CCR Model

G kinds of input vectors: *X*=(*x*_1_, *x*_2_, *x*_3_,…,*x*_*g*_)^*T*^

P kinds of input vectors: *y*=(*y*_1_, *y*_2_, *y*_3_,…,*y*_*p*_)^*T*^

CCR fractional gauge for evaluating the *j*th decision-making unit:

(2) $$\begin{array}{c} \left\{\begin{array}{c} \max\frac{u^{T}y_{0}}{v^{T}x_{0}},\\ \frac{u^{T}y_{j}}{v^{T}x_{j}}\leq 1,j=1,2,3,\ldots ,n,\\ v>0,\\ u>0, \end{array}\right. \end{array}$$

where *v* is the input index weight and *u* is the output index weight vector.

Convert formula (2) into a linear programming model:

(3) $$\begin{array}{c} \left\{\begin{array}{c} \max\mu^{T}y_{0}=h^{0},\\ s.t\;\omega^{T}x_{j}-\mu^{T}y_{j}\geq 0,j=1,2,3,\ldots ,n,\\ \omega^{T}x_{0}=1,\\ \nu \geq 0,\omega \geq 0. \end{array}\right. \end{array}$$

Reference infinitesimals *ε* make the formula more accurate and convenient:

(4) $$\begin{array}{c} \left\{\begin{array}{c} \min\left[\theta -\varepsilon \left(\sum_{e=1}^{p}s^{+}+\sum_{f=1}^{g}s^{-}\right)\right],\\ s.t.\sum_{j=1}^{n}x_{j}\lambda_{j}+s^{-}=\theta x_{0,}\sum_{j=1}^{n}y_{j}\lambda_{j}-s^{+}=y_{0},\\ \lambda_{j}\geq 0,j=1,2,3,\ldots ,n,\\ s^{+}\geq 0,s^{-}\geq 0. \end{array}\right. \end{array}$$

#### 3.2.2. BCC Model

The model is obtained by improving CCR technology [20]:

(5) $$\begin{array}{c} \left\{\begin{array}{c} \min\left[\theta -\varepsilon \left(\sum_{e=1}^{p}s^{+}+\sum_{f=1}^{g}s^{-}\right)\right],\\ s.t.\sum_{j=1}^{n}x_{j}\lambda_{j}+s^{-}=\theta x_{0,}\sum_{j=1}^{n}y_{j}\lambda_{j}-s^{+}=y_{0},\\ \sum_{j=1}^{n}\lambda_{j}=1,\\ \lambda_{j}\geq 0,\\ s^{+}\geq 0,s^{-}\geq 0,\\ j=1,2,3,...,n. \end{array}\right. \end{array}$$

#### 3.2.3. SE-DEA Model

By modifying the model [21], we can better understand the differences between efficiencies:

(6) $$\begin{array}{c} \left\{\begin{array}{c} \min\theta ,\\ s.t.\overset{n}{\underset{\begin{array}{c} j=1\\ j\neq j_{0} \end{array}}{\sum }}x_{j}\lambda_{j}=\theta x_{0},\overset{n}{\underset{\begin{array}{c} j=1\\ j\neq j_{0} \end{array}}{\sum }}y_{j}\lambda_{j}-s^{+}=y_{0},\\ \lambda_{j}\geq 0,\\ s^{-}\geq 0,\\ j=1,2,3,\ldots ,n. \end{array}\right. \end{array}$$

### 3.3. Malmquist Index

(7) $$\begin{array}{c} \text{TFP}=M\left(x^{t},y^{t},x^{t+1},y^{t+1}\right)=\text{PTEC}\times \text{SEC}\times \text{TC}, \end{array}$$

where PTEC is a pure technical efficiency change index, which measures how much of the technical inefficiency of production is caused by pure technical inefficiency. SEC is a scale efficiency change index, which is used to judge whether DMU is in the optimal production scale. TC is the change index of technological progress, which reflects the change degree of production technology.

If Malmquist >1, efficiency improved; if Malmquist <1, efficiency decreased; if it is equal to 0, it does not change. This is used to calculate the correlation efficiency index.

### 3.4. Analysis on the Present Situation of Urban Sports

Through Table 1, we know that, in the survey of this city, the number of male sports accounts for 45.5% of the total, and the number of female sports accounts for 54.5% of the total. It can be seen that women's spontaneity in sports is higher than that of men. From the perspective of sports public service, we should actively mobilize male sports enthusiasm and promote urban residents' sports.

From this Table 2, it can be seen that the age from 18 to 65 years accounts for 32.8% of the total survey, while the age under 18 years accounts for 29.5% of the total survey, and the age over 65 years accounts for 37.7%. Through the table, it is inferred that the number of sports people over 65 years old is more probable because the elderly gradually improve their health requirements and pay more attention to their health after retirement. However, the small number of sports under the age of 18 may be due to the busy school tasks. In order to pay attention to the physical health of teenagers under the age of 18, physical exercise in school should be strengthened, and only by having a healthy body can we focus more on our studies.

Through Table 3, we can see that physical education should be strengthened below junior high school. According to the table, we can infer that the higher the educational background, the greater the proportion in sports, and we have received good physical education. However, junior high school education and below pay little attention to physical exercise.

According to this Table 4, the exercise time of teenagers under 18 years old is generally 30 minutes or less, the exercise time of young adults aged 18–65 is mostly 1 hour or less, and the exercise time of elderly people over 65 years old is 1 hour or 2 hours or more. According to the analysis, teenagers under 18 years old do not have much time for sports because of their busy studies, and young adults between 18 and 65 years old cannot spare a lot of time for sports because of their busy work. Most of the elderly over 65 years old are retired people, so they can take more time to do physical exercise and strengthen their physique. In view of this situation, the urban sports public service system should increase sports venues and sports events in schools or office areas according to the study and work reasons of young adults so that people under 65 years old can easily take physical exercise after work and study.

### 3.5. Image Recognition Technology

By analyzing the accuracy and average time of the three algorithms, the accuracy and average time are obtained by randomly executing 50 times and taking the average value as shown in Table 5.

In order to reflect the performance of the algorithm, add data dimensions to analyze the accuracy and average time of image recognition in different dimensions, and the effect is shown in Figures 10 and 11.

It can be seen from the relevant data that the image recognition technology generally has high accuracy and short time, which greatly improve the efficiency of public services.

### 3.6. Improvement of Sports Public Service under Image Recognition

Through Figure 12, we know that the purpose of most investigators' sports is to enhance their physique, so urban sports public services should build related sports venues according to the purpose of enhancing people's physique. Through image recognition of people or objects, people or objects entering and leaving the gym are statistically controlled to provide residents with more comfortable and safer sports facilities in Figure 13.

In view of this trend, urban sports public service should repair more free sports venues in communities, parks, squares, and other places to provide better sports services for residents and improve their sports satisfaction so that residents can easily play sports in the vicinity of their homes in Figure 14.

According to the chart, in order to better provide urban sports public service management, square dance, runway, leisure trail, and other activity venues should be added. Cameras are installed in sports venues through image recognition to ensure the safety of residents' sports and the safety of sports venues and facilities. At the same time, professional public service management teams should be trained to compensate for the damage of manmade facilities, so as to better meet the sports needs of residents and the satisfaction of public services in Figure 15.

According to the icon, most residents study the source of sports methods by themselves. In order to provide more convenient public services, special coaches can be set up in gymnasiums to teach simple sports movements, prevent sports injuries, and improve the efficiency of urban sports public services.

## 4. Differences of Sports Public Service before and after Image Recognition

The picture of urban sports facilities under image recognition is shown in Figure 16.

Through the camera function of image recognition, urban sports facilities can be managed remotely, the damage reasons of facilities can be found out and related treatment can be carried out through image recognition, and sports personnel can also be managed by camera to ensure the safety of facilities and the sports health of residents.

It can be seen from Figure 17 that the monthly management cost of urban sports public service under the new image recognition is greatly improved compared with the traditional urban public service. The public service based on image recognition reduces the relevant management personnel, and the sports facilities and sports personnel are managed by camera through image recognition, thus reducing labor costs. In addition, when sports public facilities are damaged, we can identify whether it is manmade damage through image recognition, find the saboteurs through image recognition, and then compensate for fines, lock the faces of malicious saboteurs, and join the blacklist of sports venues.

In addition, the investment of image recognition is convenient for the management of public services and also brings convenience to the sports of urban residents. Compared with the traditional public services before, the public services under image recognition bring more people flow and enhance the sharing of community sports venues in Figure 18.

Compared with traditional public services, with the promotion of public services under image recognition. More residents choose to exercise in urban sports public services under image recognition, highlighting the improvement of public services and the convenience of residents by image recognition.

In terms of time, it takes only 2 seconds for residents to enter the public service under the venue moving image recognition to recognize faces. Traditional registration consumes several times of image recognition, almost one minute. In addition, when the flow of people is large, it is difficult to find huge data, and image recognition only needs face matching to query residents' related information.

## 5. Conclusion

According to the above research on urban sports public service based on image recognition, urban sports public service under image recognition can bring better sports service experience to residents, greatly improve residents' sports interest and facilitate residents' sports. However, there are still some drawbacks in the planning, so we should investigate the preference of men and women for sports through investigation and study, so as to promote the sports of urban residents. At the same time, according to the investigation and study of the favorite sports places or projects of residents, the improvement of urban sports venues and facilities under image recognition is carried out to better improve the efficiency of public services. According to the needs of residents' sports, we should improve the management direction of public services, create a national participation, teach residents' sports through relevant public services, and have good sports literacy to work and study actively. Improve the love of sports, reduce the harm caused by inappropriate sports, and make residents love urban sports under image recognition.

## Figures and Tables

**Figure 1:** Flowchart of image recognition.

**Figure 2:** Face recognition flowchart.

**Figure 3:** Fingerprint identification flowchart.

**Figure 4:** Classification diagram of sports facilities.

**Figure 5:** Narrow classification of sports facilities.

**Figure 6:** Planning of sports public facilities.

**Figure 7:** Influencing factors of sports public service.

**Figure 8:** Research map of sports public service of city government.

**Figure 9:** Mediation effect model diagram.

**Figure 10:** Accuracy changes with feature dimensions.

**Figure 11:** The change of feature dimension.

**Figure 12:** Table of sports goals in the survey population.

**Figure 13:** The preferred venue for physical exercise of urban residents.

**Figure 14:** Proportion of the number of people in each project.

**Figure 15:** Statistical table of motion method sources.

**Figure 16:** Sports facilities under image recognition.

**Figure 17:** Public service fee under image recognition.

**Figure 18:** Map of preferred exercise for urban residents.

**Table 1:** Sex ratio of athletes in a city survey.

Gender	Number of people	Proportion of total population (%)
Man	200	45.5
Woman	240	54.5

**Table 2:** Age ratio of athletes in a city survey.

Age	Number of people	Proportion of the total number of people surveyed (%)
Under 18 years old	180	29.5
18–65 years old	200	32.8
Over 65 years old	230	37.7

**Table 3:** Proportion of sports people's educational level in a city survey.

Education level	Number of people	Proportion of the total number of people surveyed (%)
Illiteracy	50	15.2
Primary school	55	16.8
Junior high school	43	13.1
High school	60	18.3
College degree or above	120	36.6

**Table 4:** Proportion of exercise time of athletes in a city survey.

Exercise time	Under 18 years old	18–65 years old	Over 65 years old
30 minutes or less	20	15	18
1 hour	13	17	30
2 hours and above	2	10	25

**Table 5:** Image recognition.

Image recognition algorithm	Accuracy (%)	Average time (seconds)
R-CNN [22]	53.3	13
Fast R-CNN [23]	66.0	2
Faster R-CNN [24]	73.2	1.5

## Data Availability

The experimental data used to support the findings of this study are available from the corresponding author upon request.
